# Antitumor Effect of Pseudolaric Acid B Involving Regulation of Notch1/Akt Signaling Response in Human Hepatoma Cell In Vitro

**DOI:** 10.1155/2022/5353686

**Published:** 2022-06-14

**Authors:** Haijun Gao, Yan Zhang, Xiaojin Mo, Lele Huo, Yanping Luo, Ting Zhang, Xingming Ma, Wei Hu, Tao Jing

**Affiliations:** ^1^School of Basic Medical Sciences, Lanzhou University, Lanzhou 730000, Gansu, China; ^2^National Institute of Parasitic Diseases, Chinese Center for Disease Control and Prevention (Chinese Center for Tropical Diseases Research), NHC Key Laboratory of Parasite and Vector Biology, WHO Collaborating Center for Tropical Diseases, National Center for International Research on Tropical Diseases, Shanghai 200025, China; ^3^Ganzr Tibetan Autonomous Prefecture Center for Disease Control and Prevention, Kangding 626000, Sichuan, China; ^4^National Health Commission Key Laboratory of Echinococcosis Prevention and Control, Xizang Center for Disease Control and Prevention, Lhasa 850000, Tibet Autonomous Region, China; ^5^Department of Microbiology and Microbial Engineering, School of Life Sciences, Fudan University, Shanghai, China

## Abstract

**Background:**

Liver cancer, particularly hepatocellular carcinoma (HCC), is the fourth leading cause of cancer-related death worldwide. Sorafenib is a crucial drug for the treatment of advanced HCC, but it is difficult to meet the challenge of increasing clinical demands due to its severe side effects and drug resistance. Hence, development of novel antitumor drugs is urged. Previous studies showed that pseudolaric acid B (PAB) could reduce the expression of protein kinase B (PKB/Akt), a downstream effector of Notch signaling, facilitating cell apoptosis in HCC. The disruption of Notch signaling was verified to exacerbate malignant progression and drug resistance, however, the antitumor effect of PAB on Notch signaling in HCC remains unclear. Thus, this study aims to investigate the anti-HCC effect of PAB in association with the regulation of Notch1/Akt signaling.

**Methods:**

CCK-8 assay and transwell assay were used to examine the cell proliferation and invasion in Huh7 cells after treatment with PAB and a Notch inhibitor DAPT. Moreover, the cell cycle of Huh7 cells after treatment with PAB was analyzed using flow cytometry. Finally, the changes of Notch1, Jagged1, Hes1, and Akt expression at the protein and mRNA level in Notch1/Akt signaling in Huh7 cells after treatment with PAB and DAPT were analyzed using immunofluorescence assay and real-time qPCR.

**Results:**

The proliferation rate of Huh7 cells exposed to PAB of 0.5, 1, 2, 4, 8, 10, 20, 40, 80, 100, and 200 *μ*mol/L revealed a time-and dose-dependent decrease *in vitro,* showing cell cycle arrest at G2/M phase (*P* < 0.05). Furthermore, compared with the untreated group, at the concentration of 40 *μ*mol/L, the proliferation rate and invasion rate of Huh7 cells in PAB, DAPT, and PAB-DAPT combination (PAB + DAPT) group were significantly decreased (*P* < 0.05), but the PAB + DAPT showed no synergistic antiproliferation and anti-invasion effect in comparison with PAB treatment alone (*P* > 0.05). In addition, compared with the untreated group, PAB and DAPT alone significantly downregulated the expression of Notch1, Jagged1, Hes1, Akt mRNA, or/and protein in Huh7 cells (*P* < 0.05), but there was no significant difference in synergistic downregulated effect between the PAB + DAPT group and the PAB group (*P* > 0.05).

**Conclusion:**

PAB can suppress proliferation and invasion of HCC cells through downregulating the expression of Notch1/Akt signaling protein and mRNA, and may be a potential novel antitumor drug candidate for the clinical treatment of HCC in the future.

## 1. Introduction

Liver cancer of more than 905,000 new cases causing 830,000 deaths worldwide annually is regarded as the fourth leading cause of cancer-related death worldwide [1, 2]. Among them, hepatocellular carcinoma (HCC) cases account for 90% or more, which is much higher than that of intrahepatic cholangiocarcinoma, liver angiosarcoma, and hepatoblastoma [3, 4]. It is noted that 50% or more of new cases of HCC occurs in China, of which approximately 60% are initially diagnosed as the mid or later-stage, showing a 5 year survival rate of 5%–15%, which is lower than 50%–70% of early HCC [2, 5]. At present, surgical resection, liver transplantation, and chemotherapeutics can significantly boost the treatment efficacy of early HCC, but they are difficult to meet the increasing number of patients with advanced and drug-resistant HCC [6]. Thus, some new drugs for the treatment of HCC are under development. Among them, some drugs were verified to exert strong anti-HCC effects, for example, traditional Chinese medicines [7–10], anti-inflammatory agents [11, 12], and signaling-targeting drugs [13–15]. Although sorafenib targeting tyrosine kinase receptors has been approved by the Food and Drug Administration (FDA) for the treatment of advanced HCC, based on its traits of enhancing therapeutic efficacy in most of advanced HCC patients, clinical use is limited due to its severe side effects and drug resistance [16, 17]. Therefore, it is urged to identify antitumor target molecules and develop novel drugs for HCC.

Notch signaling, a classic and conserved pathway, controls the embryonic development and tissue repairing under the physiological conditions in mammals, and contains four Notch receptors (Notch 1–4) and five ligands (Jagged−1, −2, and Delta-like−1, −3, and−4) [17, 18]. As is well known, the disruption of Notch signaling drives many pathological events in cancers, for example, malignant transformation, progression, and metastasis in colorectal cancer, pancreatic cancer, and lymphoblastic leukemia [19–21]. As well, malignant behaviors and drug resistance are closely associated with the disruption of Notch signaling in many cancers [22]; for example, the disruption of Notch signaling could facilitate epithelial-mesenchymal transition (EMT), malignant metastasis [2], and sorafenib resistance [16]. Thus, Notch signaling is a crucial diagnostic marker and drug-target in drug-resistant HCC.

Pseudolaric acid B (PAB), a traditional Chinese medicine, is a diterpene-type acid extracted from the root bark of *Pseudolarix kaempferi Gordon* and has been applied for treatment on fungal-infected dermatosis clinically for many years [23]. The previous studies suggested that PAB could block malignant behaviors in many cancers, such as driving cell apoptosis by downregulating phosphatidylinositol-3 kinase/protein kinase B (PI3 K/Akt) signaling in gastric cancer [24, 25], and inhibiting cell proliferation by blocking Akt-GSK-3*β*-catenin signaling in HCC [7]. As is well known, Akt was verified to be an important downstream effector of Notch signaling that was disrupted in sorafenib-resistant HCC [16]. However, the antitumor effect of PAB in association with the regulation of Notch/Akt signaling in HCC remains unclear and needs to be clarified. Thus, the aim of the present study was to investigate the antiproliferation and anti-invasion effects of PAB and the mechanism involving the regulation of the Notch1/Akt signaling pathway in HCC cells.

## 2. Materials and Methods

### 2.1. Biochemical Reagents

PAB, N-[N-(3, 5-Difluorophenacetyl)-L-alanyl]-S-phenyl-glycine t-butyl ester (DAPT) as a putative Notch signaling inhibitor [26], and dimethyl sulfoxide (DMSO) were purchased from Aladdin Industrial Corporation (Shanghai, China). Cell culture reagents were obtained from Gibco (Wisent, Canada). Cell Counting Kit-8 (CCK-8) kits were purchased from Beyotime Biotechnology Co., Ltd. (Shanghai, China). All used antibodies were from Cell Signaling Technology, Inc. (Bossdun, USA). The primers in polymerase chain reaction (PCR) were provided from Tsingke Biotechnology Co., Ltd. (Shanghai, China). Human hepatocyte (Huh7 cell line) was warmly presented by prof. Chen Ling from Fudan University (Shanghai, China). Extraction kits for total RNA and PCR kits were purchased from TIANGEN BIOTECH CO., LTD (Beijing, China) and Takara (Tokyo, Japan).

### 2.2. Cell Proliferation after Treatment with Drugs Assayed by CCK-8 Method

In the studies, Huh7 cell line, a liver cancer cell, was used to investigate the antitumor effect of PAB through the regulation of Notch1/Akt signaling because Huh7 cell has long been widely used to screen new anticancer drugs and explore the drug-resistant of HCC [7, 27–29]. Cell proliferation of Huh7 cells after treatment with PAB and DAPT was investigated by the CCK-8 assay and crystal violet staining. In brief, a total of 5000 and 50000 Huh7 cells per well were seeded into 96- and 24-well culture plates and incubated for 2 hours at 37°C, 5% CO_2_. Subsequently, the supernatant in the culture plates was replaced with fresh complete culture media containing 89% Dulbecco's modified Eagle's medium (DMEM), 10% foetal bovine serum (FBS), and 1% penicillin-streptomycin (P-S). At the same time, PAB at a final concentration of 0, 0.5, 1, 2, 4, 8, 10, 20, 40, 80, 100, and 200 *μ*mol/L in 0.1% DMSO, and 0.1% DMSO as the control was added into the culture plates (*n* = 8), respectively. After treatment for 24, 48, and 72 hours, Huh7 cells in the 96-well plates were reacted with CCK-8 reagents for 2 hours, and the optical density (OD) value at the wavelength of 450 nm was observed under a multifunctional enzyme marking instrument (BioTek, US), following the manufacturer's reagent instruction (Beyotime Biotechnology, Shanghai, China). Meanwhile, the Huh7 cells in 24-well plates were stained with crystal violet (Solarbio Science & Technology Co., Ltd, Beijing, China), and the cell morphology was imaged under an inverted light microscope (BX43, Olympus, Japan).

Similarly, Huh7 cells at 5000 and 50000 Huh7 cells per well were seeded into 96- and 24-well culture plates and incubated for 2 hours. Furthermore, these Huh7 cells were treated with 0.1% DMSO, 40 *μ*mol/L of PAB, 40 *μ*mol/L of DAPT, and 40 *μ*mol/L PAB plus 40 *μ*mol/L DAPT in 96-well culture plates (*n* = 8) and 24-well culture plates (*n* = 3), respectively. After treatment for 24 hours, the OD value in 96-well plates was obtained under the multifunctional enzyme marking instrument. At the same time, Huh7 cells in 24-well plates were stained with crystal violet to observe the changes in cell morphology using inverted light microscopy.

### 2.3. Examining Cell Invasion by Transwell Assay

The complete media containing different drugs was added into the bottom chambers in 24-well culture plates (550 *µ*L per well). Five experimental groups were assigned as follows: (i) the negative control (NC) group, 50 *μ*L of DMEM containing 1% P-S (*n* = 4); (ii) the vehicle or DMSO group, 50 *μ*L of 0.1% DMSO (*n* = 4); (iii) the DAPT group, treated with 40 *μ*mol/L DAPT dissolved in 0.1% DMSO (*n* = 4); (iv) the PAB group, treated with 40 *μ*mol/L PAB (*n* = 4); and (v) the PAB in combination with DAPT (PAB + DAPT) group, treated with both 40 *μ*mol/L of PAB and 40 *μ*mol/L of DAPT (*n* = 4). Furthermore, Huh7 cells in DMEM medium (5 × 10^4^ cells per well) were seeded into the upper chamber with the precoated Matrigel (BD Biosciences, San Jose, CA, USA). After treatment with drugs for 24 hours, the uninvaded Huh7 cells in the upper chamber were removed, and the invaded Huh7 cells in the lower surface of the filter were fixed with 4% paraformaldehyde and stained with 0.1% of crystal violet. Finally, the invaded Huh7 cells in three random microscopic fields per filter were imaged under a light microscope (Olympus Corporation, Tokyo, Japan), and the semiquantitative analysis of the cell invasion rate was performed by ImageJ software (National Institutes of Health, Bethesda, MD), as described previously [30]. The calculation of Huh7 cells was according to the following formula: Invasion Index = (% invasion test cell)/(% invasion control cell).

### 2.4. Examining Cell Cycle by Using Flow Cytometry

To investigate the distribution in the cell cycle of Huh7 cell after treatment with PAB, the cell cycle of Huh7 cells was measured by flow cytometry. In brief, Huh7 cells were treated with PAB 40 *μ*mol/L and untreated as the control for 24 hours and then digested with 0.25% ethylene diamine tetraacetic acid (EDTA)-free trypsin for 5 minutes. Furthermore, the collected Huh7 cells were fixed with cold 70% ethanol, followed by incubation with RNase A for 30 min at 37°C. Finally, after reacting with propidium iodide (Solarbio Science and Technology Co., Ltd., Beijing, China) for 30 min at 4°C in the dark, the cell cycle of Huh7 cells was measured under a flow cytometer (Beckman Coulter CYTOFLEX S, USA).

### 2.5. Analysis of Notch1/Akt Signaling Protein Expression by Immunofluorescence Assay

Huh7 cells (1 × 10^6^ cells per well) were seeded onto 6-well culture plates with the cell-climbing slices and then treated with the different drugs for 24 hours at 37°C, 5% CO_2,_ as described above. To assess the cell invasion by transwell assay, the experimental groups were assigned as (i) NC group (*n* = 3); (ii) DMSO group (*n* = 3); (iii) DAPT group (*n* = 3); (iv) PAB group (*n* = 3); and (v) PAB + DAPT group (*n* = 3). Thereafter, these cell-climbing slices in 6-well plates were fixed with 4% paraformaldehyde to detect the expression of Notch1 and Jagged1 proteins. Subsequently, all cell-climbing slices were blocked with 20% of normal goat serum and reacted with rabbit anti-Notch1 and Jagged1 antibodies (1 : 100 and 1 : 200) overnight at 4°C, respectively. In addition, after incubation with Cy3 and FITC conjugated goat antirabbit IgG (*H* + *L*) (1 : 200 and 1 : 500; Servicebio Technology Co., LTD., China) and DAPI (1 : 1000; Abcam, Cambridge, UK). Finally, the slides were imaged under a fluorescence microscope (Olympus, Japan), as described previously [31, 32].

### 2.6. Examination of Notch/Akt Signaling mRNA Expression by Real-Time Quantitative PCR

Similarly, after treatment with 40 *μ*mol/L PAB and 40 *μ*mol/L DAPT for 24 hours, Huh7 cells in 6-well culture plates were digested with 0.25% EDTA-free trypsin. Subsequently, collected Huh7 cells were washed with cold PBS and stored in RNAlater reagents to isolate total RNA and reverse-transcribe into cDNA. Finally, the amplification of cDNA was performed by RT-qPCR following the Takara kit protocol (No. RR036A), as described previously [33]. Notably, the following primers were used: Notch1 (forward, 5′-GGGTCCACCAGTTTGAATGG-3′; reverse, 5′-GTTTGCTGGCTGCAGGTTCT-3′), Jagged1 (forward, 5′-GGGCAACACCTTCAACCT-3′; reverse, 5′-CCAGGCGAAACTGAAAGG-3′); Hes1 (forward, 5′-TATCATGGAGAAGAGGCGAAGG-3′; reverse, 5′-TTCTCTAGCTTGGAATGCCGG-3′); Akt (forward, 5′-AGCCTGGGTCAAAGAAGTCAAAG-3′; reverse, 5′-CACAGTCTGGATGGCGGTTG-3′), and *β-actin* (forward, 5′-GGGAAATCGTGCGTGACATTAAGG-3′; reverse, 5′-CAGGAAGGAAGGCTGGAAGAGTG-3′).

### 2.7. Statistical Analysis

The experimental data are expressed as the mean ± standard deviation (SD). The group data were compared by *t*-test and unpaired comparison. Statistical analysis was performed by GraphPad Prism 8.0 (GraphPad Software, San Diego, CA) and SPSS 22.0 (IBM, Chicago, IL). *P* < 0.05 indicates significant difference.

## 3. Results

### 3.1. Analysis of Huh7 Cell Proliferation after Treatment with PAB

The CCK-8 assay showed that in comparison with the NC group, the proliferation rate of Huh7 cells was decreased in a time- and dose-dependent manner after treatment with PAB at 0.5, 1, 2, 4, 8, 10, 40, 80, 100, and 200 *µ*mol/L for 24, 48, and 72 hours. After exposure to 40 *µ*mol/L PAB for 24, 48, and 72 hours, the proliferation rate of Huh7 cells was (49.87 ± 6.99)%, (45.40 ± 3.90)%, and (2.99 ± 0.20)%, respectively, indicating that the half maximal inhibitory concentration (IC_50_) of PAB was 40 *µ*mol/L in Huh7 cells exposed for 24 hours. When the concentration of PAB was increased to 80 *µ*mol/L, the proliferation rate dramatically declined to (43.69 ± 1.36)%, (34.57 ± 0.34)%, and (2.33 ± 0.36)%, respectively (Figure 1(a)). In addition, the crystal violet staining assay revealed that in comparison with the DMSO group, a reduction in the number of Huh7 cells was recorded after treatment with 40 *µ*mol/L PAB, along with apparent cell morphological alterations, including cellular swelling and karyopyknosis (Figure 1(b)).

### 3.2. Huh7 Cell Proliferation after Treatment with PAB and DAPT

The CCK-8 assay showed that in comparison with the DMSO group [(100.00 ± 15.79)%], PAB alone or in combination with DAPT exhibited a significant decrease in the proliferation rate of Huh7 cells [(87.29 ± 6.40)% and (68.49 ± 1.16)%] (*P* < 0.0001), but there was no significant difference between the PAB group and the PAB + DAPT group (P=0.9749). Among them, the proliferation rate of Huh7 cells in the PAB group exhibited a significant decrease in comparison with that in the DAPT group [(87.29 ± 6.40)%] (*P* = 0.0010) (Figure 2(a)). In addition, the crystal violet staining assay showed that in comparison with the DMSO group, a reduction in Huh7 cell number and pathological changes of cell morphology, including swelling and karyopyknosis, were observed in Huh7 cells after treatment with PAB alone or in combination with DAPT, respectively (Figure 2(b)).

### 3.3. Analysis of Huh7 Cell Invasion after Treatment with PAB and DAPT

The cell invasion is a critical predictive risk factor in the development of HCC, thus, we investigated the anti-invasion effect of PAB on Huh7 cells by transwell assay. The results of crystal violet staining showed that after treatment with PAB or in combination with DAPT, there was a reduction in the number of Huh7 cells-invaded into matrigel layer (Figure 3(a)). Furthermore, the semiquantitative results indicated that in comparison with the DMSO group, PAB alone or in combination with DAPT exhibited a significant decrease in the invasion rate of Huh7 cells (*P*=0.0045 and *P*=0.0140), but the PAB + DAPT group did not exhibit a significant difference in comparison with the PAB group (*P*=0.9918) (Figure 3(b)).

### 3.4. Cell Cycle Arrest in Huh7 Cells after Treatment with PAB

The results of flow cytometry showed that after treatment with 40 *µ*mol/L PAB, there was an increase in the percentage of Huh7 cells at G2/M phase (Figure 4(a)). At the same time, the percentage of Huh7 cells arrested in G2/M phase after treatment with PAB was (40.84 ± 0.59)%, showing significant increase in comparison with the NC group [(6.16 ± 0.23)%] (*P* < 0.0001) (Figure 4(b)).

### 3.5. Notch1/Akt Signaling Expression at Protein Level in Huh7 Cell after Treatment with PAB and DAPT

To explore a possible antitumor mechanism of PAB on the Notch signaling pathway in HCC, the expression of Notch1 and Jagged1 were examined in Huh7 cells after treatment with PAB and DAPT. The immunofluorescence assay demonstrated that green fluorescence-stained Notch1 protein was widely distributed in the cytoplasm, not in the nuclear of Huh7 cells, but they were obviously reduced after treatment with PAB and DAPT alone, as well as their combination form, respectively. Furthermore, compared with the NC group, the expression of red fluorescence-tagged Jagged1 protein in Huh7 cells was decreased after treatment with PAB or in combination with DAPT (Figure 5).

### 3.6. Notch1/Akt Signaling Expression at mRNA Level in Huh7 Cell after Treatment with PAB and DAPT

To investigate the change of Notch1/Akt signaling at mRNA level in Huh7 cells after treatment with PAB, and the expression of Notch1, Jagged1, Hes1, and Akt mRNA were examined by RT-qPCR. The results showed that compared with the NC group, the expression of Notch1 mRNA in Huh7 cells was significantly decreased after treatment with PAB and DAPT alone (*P*=0.0031 and *P*=0.0137), as well as the PAB-DAPT combination (*P*=0.0099). Meanwhile, compared with PAB and DAPT treatment alone, no significant difference was observed after treatment with the PAB-DAPT combination (*P*=0.9279 and *P*=0.9994). Furthermore, compared with the MSO group, a significant decrease in the expression of Jagged1 mRNA in Huh7 cells was observed after treatment with DAPT and PAB alone (*P* < 0.0001 and *P* < 0.0001), as well as PAB-DAPT combination (*P* < 0.0001). In addition, we also demonstrated that PAB and DAPT alone significantly reduced the expression of Notch1 effector Hes1 mRNA in Huh7 cells, respectively (*P* < 0.0001). Similarly, the expression of Akt mRNA in Huh7 cells exposed to DAPT and PAB alone was significantly downregulated (*P*=0.0045 and *P*=0.0002), respectively, but the PAB-DAPT combination showed no significant decrease in the expression of Akt mRNA in comparison with PAB (*P*=0.8760) (Figure 6).

## 4. Discussion

Liver cancer, hepatocellular carcinoma in particular, is the fourth lethal type of cancer [1, 34]. It is generally in practice that early-stage HCC is mainly treated with surgical resection and liver transplantation, but advanced HCC requires systemic therapy, including surgical resection, liver transplantation, and drugs therapy [35, 36]. As reported, the expected 5-year survival rate of advanced HCC patients is 5%–15%. Although sorafenib has been approved for clinical treatment, the severe side effects impede its long-term use [37, 38]. Moreover, sorafenib resistance is emerging clinically, and meanwhile, it has been evidenced that the disruption of Notch/Akt signaling could drive malignant behaviors and drug resistance in many cancers [39, 40]. Thus, finding novel antitumor drugs targeting Notch/Akt signaling is a growing concern.

In this study, we found that pseudolaric acid B (PAB), a traditional Chinese medicine, could inhibit human HCC Huh7 cells proliferation in a time- and dose-dependent manner. This finding is similar to Zhang's studies that PAB exerts strong antiproliferation effect on HepG2 and SK-Hep-1 cells *in vitro* [7]. Beyond that, we found that 40 *µ*mol/L PAB exhibited a stronger inhibitory effect in Huh7 cells at (49.87 ± 6.99)% for 24 hours, indicating the IC_50_ of PAB in Huh7 cells for 24 hours is 40 *µ*mol/L. Furthermore, we also found that PAB 40 *µ*mol/L has a stronger antiproliferation effect in Huh7 cells than DAPT (a putative Notch signaling inhibitor). However, compared with PAB treatment, PAB-DAPT combination exhibited poor synergistic antiproliferation effect. Given that the cell invasion is a prerequisite for cancer metastasis in HCC [41], we investigated the anti-invasion activity of PAB on Huh7 cells. The results showed that PAB and DAPT alone could significantly suppress cell invasion in Huh7 cells. However, compared with PAB and DAPT treatment alone, treatment with PAB-DAPT combination did not show synergistic anti-invasion effect on Huh7 cells in the present study, indicating that each agent targeted different points of the same pathway to exert anti-HCC effect, of which the findings resemble that of Yang's studies [42]. Therefore, we speculate that the anti-HCC target of PAB is the same as DAPT targeting on Notch signaling. The cell cycle is regarded as a key factor regulating cell proliferation [43], our study indicated that PAB could arrest Huh7 cells in the G2/M phase, and it was reported that PAB, an antitubulin agent, can induce cell cycle arrest of tumor cells by inhibiting the aggregation of tubulin [44, 45]. In addition, PAB was evidenced to induce cell apoptosis in many cancer cells with significant increase in some proapoptotic protein expression (such as bax and cleaved-caspase-3) and significant reduction in some antiapoptotic protein expression (bcl-2) [7, 45–47]. Thus, we speculate that the proapoptotic mechanism of PAB in HCC cells may be associated with the downregulation of the antiapoptotic protein expression, and the upregulation of the proapoptotic protein expression, but which remains further verifications in future.

Furthermore, our results indicated that Notch1 protein was widely distributed in the cytoplasm of Huh7 cells, which was consistent with previous findings that Notch1 protein was mainly allocated in the cytoplasm rather than the nucleus of HCC cells [48, 49]. Moreover, we found that Jagged1, a ligand of Notch signaling, was widely presented in the cytoplasm of Huh7 cells, but it could be inhibited by PAB and DAPT (a Notch signaling inhibitor), resulting in a significant reduction in the expression of Notch1 protein. More importantly, in our studies, PAB-DAPT combination treatment showed no synergistic downregulation effect on both Jagged1 and Notch1 protein expression in Huh7 cells when compared with PAB and DAPT treatment alone. The expression of Notch1 and Jagged1 mRNA in Huh7 cells were also significantly downregulated by treatment with PAB and DAPT alone, but PAB-DAPT combination did not exhibit synergistic downregulation on mRNA expression, which supported the previous hypothesis that antiproliferation and anti-invasion effect of PAB were processed by suppressing Notch1/Jagged1 signaling. Furthermore, it was found that no additive inhibitory effect was detected by some drug combinations, suggesting that each agent targeting different levels of the same pathway may result in a full effect [42]; however, other studies argued that synergistic effect of some drugs may be triggered by targeting the same signaling pathway [50]. Notch signaling is activated after the ligand binds to an adjacent Notch receptor in the neighboring cells. The expression of hairy and enhancer of split 1 (Hes1), a Notch target gene, could be upregulated to trigger the downstream signal transduction [22, 51]. The present study demonstrates that the expression of Hes1 mRNA was significantly downregulated after treatment with PAB and DAPT alone in Huh7 cells, but not with the PAB-DAPT combination.

Akt is often regarded as an important downstream effector of Notch signaling [16]. It was evidenced that the PI3K/AKT signaling pathway could be inhibited by PAB in gastric cancer cells [25]. Corroborating the previous findings, our study found that PAB and DAPT alone could significantly reduce the expression of Akt mRNA, but the PAB-DAPT combination did not.

Taken collectively, our results suggested the mechanism of PAB inhibiting the proliferation and invasion of human HCC cells by downregulating Notch1/Jagged1/Hes1/Akt signaling cascades. However, the potential antitumor effect of PAB on HCC needs to be verified. In addition, several studies have suggested that PAB can relieve drug resistance in gastric cancer and breast cancer [46, 52]. Meanwhile, sorafenib resistance in HCC is closely associated with the disruption of Notch signaling [22], and apoptosis cell death in cancer cells is also closely associated with Notch signaling [53]. Therefore, to investigate how PAB reverses drug resistance and boosts apoptosis of HCC cells through the regulation of the Notch1/Akt signaling pathway is currently in progress in our group.

## 5. Conclusions

PAB could inhibit proliferation and invasion of human hepatoma carcinoma Huh7 cells and arrest the Huh7 cell at G2/M phase, which were processed by downregulating the expression of Notch1/Akt signaling, and PAB may be a promising antitumor candidate drug for the clinical treatment of HCC.

## Figures and Tables

**Figure 1:** Antiproliferation effect of PAB on Huh7 cell. (a) The proliferation rate of Huh7 cells exposed to PAB of 0.5, 1, 2, 4, 8, 10, 20, 40, 80, 100, and 200 *μ*mol/L for 24, 48, and 72 hours, as measured by CCK-8 assay. (b) The Huh7 cell morphology exposed to 40 *µ*mol/L of PAB for 24 hours, as measured by crystal violet staining assay. Scale-bars: 100 *μ*m.

**Figure 2:** Antiproliferation effect of PAB and DAPT on Huh7 cell. (a) The proliferation rate and (b) Huh7 cell morphology exposed to PAB and DAPT of 40 *μ*mol/L for 24 hours, as measured by CCK-8 assay and crystal violet staining assay. Data are expressed as mean ± SD, *n* = 8. ^*∗*^*P* < 0.05, ^*∗∗∗*^*P* < 0.001, ^*∗∗∗∗*^*P* < 0.0001. Scale-bars: 100 *μ*m. ns, no significance.

**Figure 3:** Anti-invasion effect of PAB and DAPT on Huh7 cell. (a) The cell morphology and (b) the invasion of Huh7 cell after treatment with PAB and DAPT of 40 *μ*mol/L for 24 hours, as measured by crystal violet staining assay and transwell assay. Data are expressed as mean ± SD, *n* = 4. ^*∗*^*P* < 0.05, ^*∗∗*^*P* < 0.01. Scale-bars: 100 *μ*m. ns, no significance.

**Figure 4:** The cell cycle arrest in Huh7 cell after treatment with PAB. (a) The distribution of Huh7 cells cycle after treatment with 40 *μ*mol/L PAB for 24 hours, as measured by flow cytometry, and (b) the semiquantitative analysis of the cell cycle arrest of Huh7 cell. Data are expressed as mean ± SD, *n* = 3. ^*∗∗∗∗*^*P* < 0.0001.

**Figure 5:** The expression of Notch1 and Jagged1 protein in Huh7 cell after treatment with 40 *μ*mol/L PAB and of 40 *μ*mol/L DAPT for 24 hours, as detected by immunofluorescence assay. Scale bars: 20 *μ*m.

**Figure 6:** The expression of Notch1, Jagged1, Notch effector Hes1, and Akt mRNA in Huh7 cells after treatment with both 40 *μ*mol/L PAB and 40 *μ*mol/L DAPT for 24 hours, as detected by RT-qPCR. Data are expressed as mean ± SD, *n* = 3. ^*∗*^*P* < 0.05, ^*∗∗*^*P* < 0.01, ^*∗∗∗*^*P* < 0.001, and ^*∗∗∗∗*^*P* < 0.0001.

## Data Availability

These data that are used or analyzed in the research can be obtained from the corresponding author according to reasonable requirements.
